# Current Progress on Neuroprotection Induced by Artemisia, Ginseng, Astragalus, and Ginkgo Traditional Chinese Medicines for the Therapy of Alzheimer's Disease

**DOI:** 10.1155/2022/3777021

**Published:** 2022-06-14

**Authors:** Qin Li, Limor Rubin, Marta Silva, Shuai Li, Chao Yang, Philip Lazarovici, Wenhua Zheng

**Affiliations:** ^1^Center of Reproduction, Development and Aging and Institute of Translation Medicine, Faculty of Health Sciences, University of Macau, Taipa, Macau 999078, China; ^2^College of Pharmacy, Hangzhou Medical College, Hangzhou, Zhejiang, China; ^3^Allergy and Clinical Immunology Unit, Department of Medicine, Hadassah-Hebrew University Medical Center, Jerusalem 9112001, Israel; ^4^MoE Frontiers Science Center for Precision Oncology, University of Macau, Macau SAR, China; ^5^Guangdong Provincial Key Laboratory of Biomedical Imaging, The Fifth Affiliated Hospital, Sun Yat-sen University, Zhuhai, China; ^6^Pharmacology, School of Pharmacy Institute for Drug Research, Faculty of Medicine, The Hebrew University of Jerusalem, Jerusalem 9112002, Israel

## Abstract

Aging is associated with the occurrence of diverse degenerative changes in various tissues and organs and with an increased incidence of neurological disorders, especially neurodegenerative diseases such as Alzheimer's disease (AD). In recent years, the search for effective components derived from medicinal plants in delaying aging and preventing and treating neurodegenerative diseases has been increasing and the number of related publications shows a rising trend. Here, we present a concise, updated review on the preclinical and clinical research progress in the assessment of the therapeutic potential of different traditional Chinese medicines and derived active ingredients and their effect on the signaling pathways involved in AD neuroprotection. Recognized by their multitargeting ability, these natural compounds hold great potential in developing novel drugs for AD.

## 1. Introduction

Aging is associated with an accumulation of several detrimental changes in cells, tissues, and organs that affect the body's normal functioning and increase the risk of disease and death. Over the years, the increase of life expectancy brought to central stage concerns related to the increase of aging-associated chronic neurodegenerative diseases, such as Alzheimer's disease (AD). AD, the most common cause of dementia, is a complex, multifactorial, and progressive neurodegenerative disease, affecting about 5% of the population over 65 years old that accounts for 60-80% of the total number of AD patients [1, 2]. According to AD International data, there are currently 46.8 million AD patients in the world, and with the increase of the aging population, this incidence is expected to continue rising to nearly 131.5 million by 2050, posing a significant economic burden to society and caregivers [3].

AD main pathological features include diffuse brain atrophy, the extracellular accumulation of amyloid plaques composed of A*β* protein, the presence of intracellular neurofibrillary tangles (NFTs) composed of hyperphosphorylated microtubule-associated tau protein, and extensive neuronal loss [4]. These changes occur gradually impairing the patients' cognitive functions affecting memory, learning, speech, and judgement. As the disease progresses, AD pathological changes become more pronounced severely affecting ability of patients to perform basic functions and ultimately leading to death [5]. Despite the multitude of proposed hypotheses to explain the etiology and pathology of AD and the considerable medical progresses made in the last 30 years, AD pathophysiological mechanisms are still unclear, hampering the development of effective therapeutic approaches [6]. Currently approved therapies include cholinesterase inhibitors (donepezil, galantamine, and rivastigmine), the N-methyl-D-aspartate (NMDA) receptor (NMDAR) antagonist memantine, and, more recently, aducanumab that is a monoclonal antibody that targets A*β* aggregates in the brain. Nevertheless, these drugs provide only a temporary symptomatic relief, failing to improve the patients' cognitive function or to provide a definitive cure [7].

In recent years, the use of different medicinal plant-derived products and supplements has increased greatly, with a large population relying on them as complementary and alternative to primary healthcare medicines [8]. In China and other Asian countries, traditional Chinese medicines (TCMs) have long been used for the prevention and treatment of neurodegenerative diseases. In line with this trend, during the past few years, an increasing number of publications reported the beneficial therapeutic effects of different medicinal plants on the improvement of AD symptoms in animal models and patients, with few adverse effects [9–13]. Compared with other drugs, medicinal plants represent potent, multitarget agents for the treatment of neurological disorders with relatively good efficacy, safety, and cost-effectiveness [14]. Therefore, the development of innovative anti-AD compounds derived from medicinal plants such as TCM may become an effective alternative approach for the treatment of AD [15–18]. This review provides an overview of selected traditional Chinese plant extracts and derived active ingredients, reported to have good clinical tolerability, that affect important protein targets in AD pathology and beneficially modulate several cellular signaling pathways towards correction of pathologies in AD therapy.

## 2. Neuroprotection towards Programmed Cell Death Induced by A*β* and Tau Protein Misfolding in AD

A*β* peptides derive from the sequential cleavage of amyloid precursor protein (APP), induced by the *β*-site APP cleaving enzyme1 (BACE1) and *γ*-secretase [19]. According to the amyloid cascade hypothesis, AD pathophysiology is primarily due to the aggregation of A*β* misfolded oligomer peptides [20], triggered by an imbalance between A*β* production and clearance [21], that ultimately impairs neuronal and synaptic function and induces cell death. *γ*-Secretase is a complex transmembrane protease comprised of nicastrin (NCSTN), presenilin (PEN-1), anterior pharynx-defective 1 (APH-1), and presenilin enhancer 2 (PEN-2) subunits that can be potentially targeted to modulate A*β* production and clearance [22, 23]. Thus, both BACE and *γ*-secretase enzymes have been pursued as potential targets to modulate A*β* production upstream in the amyloid cascade. Under normal physiological conditions, tau protein is a microtubule-associated protein that stabilizes neuronal microtubules. However, in AD, tau protein has been found in a hyperphosphorylated state forming aggregates of paired helical filaments and misfolded neurofibrillary tangles (NFTs) that compromise both neuronal and synaptic functions [24]. The accumulation of conformational changes and protein misfolding has been widely correlated with the induction of endoplasmic reticulum (ER) stress that ultimately leads to neuronal dysfunction and cell death [25, 26]. Therefore, preventing the misfolding or aggregation of A*β* peptides or hyperphosphorylated tau protein has been proposed as a potential approach to target AD pathogenesis [27].

The occurrence of abnormalities in programmed cell death (PCD) pathways, which are crucial signaling events occurring during normal neuronal development of the central nervous system, has been commonly described in neurodegenerative diseases such as AD. The abnormal activation of PCD events, such as apoptosis, necroptosis, pyroptosis, autophagic cell death, and necrosis, has been reported in the pathogenesis of AD [28]. Apoptosis is mainly triggered by the intrinsic and the extrinsic pathways that promote the activation of caspase proteases [29]. The intrinsic pathway is a mitochondrial-mediated pathway that can be triggered by insults such as oxidative stress and that is regulated by BCL-2 family members of antiapoptotic proteins [30]. The extrinsic pathway is a death receptor-mediated pathway that can be triggered upon the attachment of death ligands, such as tumor necrosis factors (TNF), to the extracellular domain of the death transmembrane receptors [31]. In AD, caspase activation and mediated cleavage of APP have been closely associated with the occurrence of synapse loss [32]. Moreover, evidence suggest that A*β* accumulation promotes apoptosis through the upregulation of the cell death effector BAX and downregulation of the antiapoptotic proteins BCL-2 and BCL-XL levels [33]. Recent research has confirmed the accumulation of A*β*_1-42_ in some degenerating-shape neurons in AD cases, suggesting that the A*β*_1-42_ pathway may be directly relevant to neuronal loss in AD [34]. Similar studies have found that microinjection of A*β*_1-42_ peptide or a cDNA-expressing cytosolic A*β*_1-42_ rapidly induces cell death of primary human neurons and confirmed that intracellular A*β*_1-42_ is selectively cytotoxic to human neurons through the p53/Bax cell death pathway [35].

Necroptosis, another form of regulated cell death, is characterized by cytoplasmic swelling (oncosis), loss of plasma membrane integrity, swelling of cytoplasmic organelles, formation of the necrosome complex in the cytosol, ROS production, and release of damage-associated molecular patterns (DAMPs) that may ultimately drive inflammation [36, 37]. Different studies have confirmed the occurrence of necroptosis with inflammasome activation and increased IL-1*β* and IL-18 levels in AD [38–41]. Current research indicated that an antinecroptotic molecule named necrostatin-1 (Nec-1) directly targets A*β* and tau proteins, alleviates brain cell death, and ameliorates cognitive impairment in AD models [42]. Therefore, alleviation of neural cell death is as an important goal in AD therapy, representing a promising avenue to be explored in TCM-induced AD therapy.

TCM contains multiple phytochemicals that have a general neuroprotective effect and therefore may prove beneficial in different neurodegenerative disorders [43]. Neuroprotection in AD refers to mechanisms and strategies that are aimed at protecting the nervous system from injury and damage to slow down, prevent, or stop PCD during degeneration and thus restoring the function of the damaged neuronal pathways [44]. Many of the medicinal plants with neuroprotective and antineurodegenerative potential belong to plant families such as *Compositae*, *Labiaceae*, *Ranunculaceae*, and *Zingiberaceae*. This review will explore the potential of a few selected TCMs in reducing misfolding of A*β* and tau proteins and conferring neuroprotection towards PCD, by focusing on preclinical and clinical research progress achieved on *Artemisia annua*, *Ginseng*, *Astragalus membranaceus*, and *Ginkgo biloba* leaf extract and derived chemicals as anti-AD compounds using *in vitro* neuronal cell cultures, *in vivo* animal models of AD, and selected few clinical trials.

### 2.1. *Artemisia annua*

Artemisinin is a sesquiterpenoid complex extracted from the traditional Chinese herb *Artemisia annua* that has been used as a first-line antimalarial drug in the clinic for decades, saving the lives of millions of people [45]. Characterized by a molecular formula of C_15_H_22_O_5_, it contains an endoperoxide 1,2,4-trioxane ring that is critical for its pharmacological activities [46, 47]. Since its first isolation, several other Artemisinin analogs have been developed, such as Dihydroartemisinin (DHA), Artemether, Arteether, and Artesunate (Figure 1(a)), that have improved solubility and pharmacokinetic profiles [48–50].

Artemisinin and its derivatives are characterized by a high efficacy, affordability, and excellent capability to cross the blood-brain barrier (BBB) and proven safety [51]. Over the years, the research performed on these antimalarial compounds provided evidence of a wide range of other pharmacological actions [52]. In particular, we and others have recently found that Artemisinins exhibit important neuroprotective effects [53–57]. For example, in vitro studies showed that Artemisinin and derivatives confer neuroprotection towards PCD as they are able to protect PC12 and SH-SY5Y cells, primary cortical and hippocampal neuronal cultures, and human retinal pigment epithelial D_407_ cells, exposed to sodium nitroprusside (SNP), hydrogen peroxide (H_2_O_2_), and A*β* insults [54–57]. In addition, Artemisinin and derivatives also improved learning and memory impairments and corrected some pathological alterations such as A*β* deposition in different AD experimental mouse models [58–60]. Further analysis showed that Artemisinin and Artemether neuroprotective action in 3xTg AD mice occurred by stimulation of the ERK/AMPK/GSK3(ser9)/Nrf2 signaling pathways [59, 60]. The derivative Artesunate was also shown to significantly decrease A*β* formation by inhibiting the amyloid precursor protein- (APP-) cleaving enzyme 1 (BACE-1) in BV2 mouse microglia-derived cell cultures exposed to lipopolysaccharide (LPS) insults [61–63]. Artemether also attenuated A*β*_25-35_-induced cognitive impairments by downregulating A*β*, BACE1, and tau proteins in a rat model [64]. These findings, combined with the fact that Artemisinins can easily cross the BBB, highlight their potential as therapeutic candidates for the treatment of neurodegenerative disorders such as AD [65]. However, the assessment of the therapeutic potential of Artemisinin and its analogs towards age-associated neurodegenerative diseases is still in an early stage [66].

### 2.2. *Ginseng*

Ginseng (*Panax ginseng* C. A. Meyer) is a perennial herb of the Araliaceae family whose dried roots have been traditionally used as medicine in Asia. Ginsenosides, the main constituents and major active ingredients of ginseng, represent a class of steroid glycosides and triterpenoid saponins [67]. These compounds have a four-ring steroidal structure with attached sugar moieties (Figure 1(b)) that account for their pharmacological activities by enabling their interaction with cell membranes, ion channels, and receptors [68]. Depending on the position and amount of sugar moieties, ginsenosides can be divided into A-panaxadiol group (Rb1, Rb2, Rb3, Rc, Rd, Rg3, and Rh2), B-panaxatriol group (Re, Rg1, Rg2, and Rh1), and C-oleanolic acid group (Ro) [69]. In recent years, the neurotrophic and neuroprotective effects of ginsenosides in neurodegenerative diseases such as AD, Parkinson's disease, and vascular dementia have attracted much attention [70, 71]. For example, patients with moderately severe AD, treated with ginseng powder, showed significant improvement in their cognitive function [72]. Ginsenoside Rg1 repaired hippocampal long-term potentiation and memory in an APPswe/PSEN1dE9 AD mouse model, in correlation with reduced astrocyte activation and increased proliferation of the hippocampal cells. Ginsenoside Rg1 upregulates the mRNA expression and secretion of glial cell-derived neurotrophic factor (GDNF), brain-derived neurotrophic factor (BDNF), and nerve growth factor (NGF) [73]. Ginsenoside Rb1 stimulated Schwann cell proliferation and increased the expression and secretion of both NGF and BDNF [74]. Moreover, ginsenosides (Rb1, Rb2, Rc, Re, Rg1, and Rg3) act through inhibition of AChE, BChE, and BACE1 activities, as well as scavenging of ONOO(-) and inhibition of nitrotyrosine formation, to treat or prevent Alzheimer's disease [75]. Previous studies reported that the decrease of the neurotrophin BDNF level is related to the onset of AD [76]. Reduced levels of BDNF in the hippocampus of AD patients were found to correlate with the apoptosis and degeneration of cholinergic neurons [77]. The latest research also confirmed that the BDNF gene therapy was a promising method for the treatment of AD according to a phase I clinical trial of aav2-BDNF gene therapy for early Alzheimer's disease and mild cognitive impairment, which protects against tau-related neurodegeneration of Alzheimer's disease [78]. Interestingly, similar studies have confirmed ginsenoside Rg1's ability to upregulate BDNF expression, proof of concept that may serve as another therapeutic approach for AD [79]. Ginsenoside Rd was also reported to improve the learning and memory deficits in a rat model of AD, upon bilateral injection in the hippocampus with A*β*_1-40_. Ginsenoside Rd promoted the downregulation of caspase-3 proteins and therefore contributed to the reduction of apoptosis [80]. In conclusion, *Panax ginseng*, a well-known medicinal plant that contains ginsenosides, gintonin, and other components, has neuroprotective effects in neuronal cells and animal models by stimulation of BDNF expression in AD. The findings from clinical trials further indicate that *Panax ginseng* or its formula treatment is safe and has a positive effect on cognition in patients with AD [81–83]. Therefore, it is of great value to carry out clinical trial research to further evaluate the therapeutic effects of ginseng, formulas, and combinations with other TCM and drugs, in patients with different stages of AD, and further explore the underlying molecular mechanisms of neuroprotection [84].

### 2.3. *Astragalus membranaceus*

*Astragalus membranaceus* is a medicinal herb from the Fabaceae/Leguminosae family commonly used in several herbal formulations of TCM and containing complex bioactive components, including flavonoids, saponins, and polysaccharides [85]. Astragaloside IV (AS-IV) (Figure 1(c)), a small molecular saponin purified from *Astragalus membranaceus* [86], is the main active ingredient and is well-known for its multiple peripheral pharmacological effects and central nervous system neuroprotective effects [87–89], with evidences in animal models indicating its therapeutic potential for AD [90–92] and Parkinson's disease (PD) [93–95]. For example, Costa et al. performed a systematic review on the neuroprotective effects induced by AS-IV in experimental models of neurological disorders covering the years between 2007 and 2017 and pointed to the fact that administration of AS-IV can improve behavioral and neurochemical deficits largely due to its antioxidant, antiapoptotic, and anti-inflammatory properties [90].

Similar research findings indicated that Astragalus extract can significantly improve the learning and memory abilities of AD mice and downregulate caspase-3 mRNA levels, decrease the expression of the caspase-3 protein and cytochrome c in the hippocampus and neocortex, and inhibit caspase-9 and caspase-3 activities [96]. AS-IV treatment reduced cortical neuron degeneration and memory deficits in AD rats and inhibited A*β*-induced PD. [97] Furthermore, evidence was provided on the ability of AS-IV to promote neural stem cell (NSC) differentiation in the AD rat model [98]. Specifically, grafting of AS-IV-treated NSCs into the hippocampus of AD rats improved learning and memory skills, by stimulating NSC proliferation and differentiation, partly by the Notch signaling pathway [99]. In phase I clinical trial, the safety and tolerance of Astragaloside injection (AGI) were investigated in 62 healthy volunteers. It was found that the maximum tolerance is 600 mL for single-dose treatment and 400 mL for multiple-dose treatment (7 days) [100]. .The dose guidance given in this study allows, and calls, for examination in patients with Alzheimer's disease in a phase II clinical trial. Interestingly, a similar clinical study performed in China indicated that AS-IV enhances stroke patients' recovery from their neurological disability and improves functional outcome [101].

### 2.4. *Ginkgo biloba* Extracts

Extracts from *Ginkgo biloba* leaves have been long used as supplements for the treatment of neurodegenerative dementias associated with aging, Parkinson's, and Alzheimer's due to its beneficial effects on cognition, memory, and neuronal plasticity [102]. EGb761 (*Ginkgo biloba* extract EGb761-Rökan, Tanakan, Tebonin) is a standardized extract of Ginkgo biloba leaves that has antioxidant properties as a free radical scavenger and is a well-defined product that contains approximately 24% flavone glycosides and 6% terpene lactones. Ginkgolide B and bilobalide account for about 0.8% and 3% of the total extract, respectively. Other constituents include proanthocyanadins, glucose, rhamnose, organic acids, D-glucaric, and ginkgolic acids. EGb761, which was originated by Schwabe Pharmaceuticals Co., has been available in Europe as a herbal extract since the early 1990s. However, products containing EGb761 are not approved for use by the USA-FDA. As a dietary supplement, Nature's Way in the USA distributes and markets a standardized extract of Ginkgo biloba leaves (the EGb761 formula) under the name Gingold Nature's Way [103, 104]. Numerous studies have been performed to evaluate the neuroprotective effect of EGb761 with shreds of evidence suggesting clinical efficacy in the treatment of cognitive deficits in age-associated memory disorders [105]. Treatment of a transgenic Tg2576 AD mouse model with EGb761 significantly enhanced spatial learning and memory skills. Evidence that EGb761 can lower the circulating free cholesterol levels, thereby inhibiting the production of A*β* and amyloid precursor protein (APP), has also been reported [106]. Interestingly, the *Ginkgo biloba* extracts are also able to reduce the A*β* toxicity by inhibiting the formation of A*β*-fibrils [107]. Recently, ginkgolide A (but not B and C), bilobalide, and flavonoids (Figure 1(d)) were found to enhance the PCD autophagic activity and degradation of the phosphorylated-cytoskeleton tau protein in the lysosomes of neurons [108]. In addition, *Gingko biloba* extract was found to improve cognitive function, decrease phosphorylated-tau protein levels, and ameliorate the loss of synaptophysin in tau-transgenic mice and neuronal cultures [97]. The beneficial effect of EGb761 on synaptic function and neuronal plasticity has also been investigated in hippocampal neurons [109]. MEDLINE, Cochrane, and other relevant databases were searched in March 2014 for eligible randomized controlled trials of Ginkgo biloba-EGb761 therapy in patients with cognitive impairment and dementia, and nine trials met the inclusion criteria. Clinical trials were of 22-26-week duration and included 2,561 patients. In the meta-analysis, the weighted mean differences in change scores for cognition were in favor of EGb761 compared to placebo; the standardized mean differences in change scores for activities in daily living were also in favor of EGb761 compared to placebo and showed a statistically significant difference from placebo using the Clinicians' Global Impression of Change (CGIC) scale, used to quantify and track patient progress and treatment response over time. Finally, safety data revealed no important safety concerns with EGb761 and a dose of 240 mg/day stabilized or slowed the decline in cognition, function, behavior, and global change at 22-26 weeks in cognitive impairment and dementia, especially for patients with neuropsychiatric symptoms [110]. Mild cognitive impairment (MCI) is a neurocognitive state between normal cognitive aging and dementia, with evidence of neuropsychological changes but insufficient functional decline to ensure diagnosis of dementia. Individuals with MCI are at increased risk for progression to dementia, and a significant proportion display neuropsychiatric symptoms, also a known risk factor for dementia. On the other hand, cerebrovascular disease (CVD) is thought to be a known risk factor for MCI/dementia. The Ginkgo biloba extract, EGb761, is increasingly being used for the symptomatic treatment of cognitive disorders with and/or without CVD, due to its known neuroprotective effects and cerebrovascular benefits. The ASian Clinical Expert group on Neurocognitive Disorders (ASCEND) critically assessed the current evidence on the general management of MCI, including the efficacy and safety of EGb761 as a treatment option in MCI. EGb761 has demonstrated symptomatic improvement in at least four randomized trials, in terms of cognitive performance, memory, recall and recognition, attention and concentration, anxiety, and NPS. There was also evidence that EGb761 delayed progression from MCI to dementia in some individuals. This expert group suggested that it is clinically appropriate to incorporate EGb761 as part of the multiapproach intervention for MCI [111]. Furthermore, a full understanding of the neuroprotective mechanisms of action of *Ginkgo biloba* extracts is still required to fully accomplish its clinical potential in the therapy of neurodegenerative diseases such as AD.

## 3. Modulation of Cholinergic and Glutamatergic Neurotransmission in AD

Impairments in glutamatergic and cholinergic neurotransmission, which are involved in learning and memory processes, are associated with pathological changes responsible for the clinical symptoms observed in AD. Dysfunction in the glutamatergic system by A*β* oligomers induces N-methyl-d-aspartate- (NMDA-) dependent calcium Ca^2+^ overload in the postsynaptic neurons, generating a slow excitotoxicity process, followed by neuronal oxidative stress that may lead to direct impairment of cognition and, in the long term, neuronal loss [112]. A*β* peptides have also been shown to depress the release, synthesis, and axonal transport of acetylcholine [113]. Cholinergic dysfunction in the forebrain is associated with early cognitive impairments observed in AD, correlates with cognitive decline, and forms the basis of the “cholinergic hypothesis” of AD [114]. The two drug classes currently available for the treatment of AD are the noncompetitive NMDA receptor antagonist, memantine, that normalizes dysfunctional glutamatergic neurotransmission, and acetylcholinesterase inhibitors (donepezil, galanthamine, and rivastigmine) which increase synaptic ACh levels [115]. As monotherapies, these drug types have demonstrated significant symptomatic efficacy in AD, and existing clinical data suggest that their combined use may bring additional benefit [116]. With this background, it was reported that TCM extracts [117] and derived flavonoids, alkaloids, ketones, polyphenols, terpenoid, and saponin constituents [118] inhibit acetylcholinesterases and glutamate signaling [119].

Oil of flower *Artemisia annua* has acetylcholinesterase (AChE) inhibitory activity [120]. Notoginsenoside R1 increased choline acetyl transferase expression thereby increasing acetylcholine level, in an APP/PS1 double-transgenic mouse model of AD as compared to the vehicle-treated mice [121]. Polyacetylene compounds in hexane and methanol extracts of ginseng were reported to inhibit AChE [122], and wild ginseng root extract (HLJG0701-*β*) inhibited AChE *in vitro* and *in vivo* [123]. Ginsenosides F1, Rd, Rk3, 20(S)-Rg3, F2, and Rb2 were found to possess strong AChE inhibitory activities [124]. Ginsenosides Rb1, Rb2, Rc, Re, Rg1, and Rg3 have significant inhibitory potential against AChE and butyrylcholinesterase (BChE), explaining their antineurodegenerative benefits similar to the AChE inhibitors in Alzheimer's therapy [125]. Six major compounds, namely, calycosin-7-O-*β*-d-glucoside, pratensein-7-O-*β*-d-glucoside, formononetin-7-O-*β*-d-glucoside, calycosin, genistein, and formononetin, with AChE-binding affinities were identified and isolated from the *Astragalus membranaceus* extracts [126]. Standardized extracts of *Ginkgo biloba* showed a dose-dependent inhibitory effect on AChE activity *in vitro* [127] and *in vivo* [128]. Ginkgolide B significantly inhibited AChE activity and enhanced the activity of choline acetyltransferase (ChAT) in A*β*_25–35_-treated cholinergic nerves in the rat hippocampus [129].

Artemisinin analog *α*/*β* Arteether at 25-50 mg/kg for two days of treatment decreased the NMDAR expression in mice [130]. Ginsenoside Rg3 protects NMDA-induced neuronal death via competitive interaction with the glycine-binding site of NMDA receptors in cultured hippocampal neurons [131], and ginsenoside Rk1 inhibited NMDARs most effectively among the five compounds (Rg3, Rg5, Rk1, Rg5/Rk1 mixture, and protopanaxadiol) on cultured hippocampal neurons by an interaction with the polyamine-binding site of the NMDAR channel complex [132]. Ginsenoside Rd inhibited in vivo the hyperphosphorylation of NR2B subunit and decreased its expression levels [133]. Astragaloside IV or saponins extracted from *Astragalus* decreased the level of glutamate (Glu), glutamine (Gln), glutaminase (GA), and glutamine synthetase (GS) in different brain regions of male rats [134]. EGb761 and its monomer component ginkgolides inhibited the postischemic LTP, by inhibiting the EPSCs and the *α*-amino-3-hydroxy-5-methyl-4-isoxazole propionic acid (AMPA) subtype of glutamate receptor subunit GluA1 expression on postsynaptic rat hippocampus membrane [135], and ginkgolide A inhibited NMDA receptors in mouse primary cortical neurons [136]. Cumulatively, these findings indicate that the TCM discussed in this review correct cholinergic and glutamatergic neurotransmission, like the AChE inhibitors and memantine drugs used in the clinic.

## 4. Neuroprotection towards Calcium Overload, Oxidative Stress, and Mitochondrial Dysfunction in AD

Calcium overload, mitochondrial dysfunction, and oxidative cell injury induced by misfolded tau and *β*-amyloid play an important role the pathological changes seen in AD [137]. Under normal physiological conditions, neuronal and glial cells use calcium regulatory protein tools to maintain Ca^2+^ homeostasis. Intracellular Ca^2+^ level is determined by a balance between the calcium channels and extruder proteins. Key components in regulating calcium homeostasis in cells include the sodium/calcium exchanger (NCX) and plasma membrane calcium-ATPase (PMCA) which actively remove Ca^2+^ from the cells and sarcoendoplasmic reticulum calcium-ATPase (SERCA) that sequesters this cation in the endoplasmic reticulum (ER) [138]. In AD pathologic conditions, excessive entry of Ca^2+^ into the cytoplasm and thereafter into the mitochondria triggers calcium release from the mitochondria, which in turn induces further calcium release by mitochondrial Ca^2+^-induced Ca^2+^ release [139]. Moreover, the pathological increase in intracellular calcium level, defined as calcium overload, is a multiphasic gradual process that includes besides mitochondrial calcium also Ca^2+^ ions released from the ER as well as extracellular influx across the plasma membrane. Oxidative stress is defined as an increase over physiologic values of the intracellular concentration of reactive oxygen species (ROS). These ROS are free radicals containing one or more unpaired electrons which can damage many macromolecules and cell structures. Mitochondria are a very important endogenous source of ROS. The imbalance between prooxidative and antioxidant capacity (redox potential) has been confirmed to represent an important pathological event in AD.

### 4.1. Decreased Calcium Overload

With this background, it is important to stress the ability of the different TCMs to reduce the calcium overload (Figure 1(e)) by different mechanisms. Chloroform extract of *Artemisia annua* fully abolished voltage-dependent Ca^2+^ channel (VDCC) currents [140]. Both the depolarization and the repolarization of the nerve action potentials were markedly inhibited by Artemisinin in a concentration- and time-dependent manner in either A-type or C-type nodose ganglion neurons [141]. Ginseng total saponins and ginsenosides Rf and Rg3 conferred neuroprotective effects towards L-type Ca^2+^channel-mediated cell death in rat cortical neurons [142]. Ginsenosides Rg3 and Rh2 are the major inhibitors of voltage-dependent calcium channels in *Panax ginseng*, and they show some calcium channel subtypes selectivity [143]. Ginsenoside Rd inhibited L-type calcium current in patch-clamp experiments [144], and ginsenoside Rb1 selectively inhibited the activity of L-type voltage-gated calcium channels in cultured rat hippocampal neurons [145]. Astragaloside IV affected Ca homeostasis through two opposite pathways: inhibition of Ca influx through L-type Ca channel and promotion of Ca release from sarcoplasmic reticulum [146]. Cumulatively, these actions may reduce the calcium overload in AD-insulted neurons, therefore conferring neuroprotection.

### 4.2. Inhibition of the Oxidative Stress

Oxidative stress is widely recognized as a critical component of the pathogenesis and progression of AD. For example, the Butterfield laboratory discovered the oxidative stress associated with oligomeric amyloid-*β* peptide manifested primarily as elevated oxidative modification of proteins and peroxidation of lipids. This oxidative damage caused neuronal death, which significantly underlies the progressive loss of cognition in AD [147]. Albeit mitochondria regulate cellular levels of ROS, they cannot remove all radicals produced during AD insult. SOD is considered to be the first line of defense against excess free radicals by catalyzing the conversion of the superoxide radical to hydrogen peroxide with the simultaneous production of oxygen. This facilitates the spontaneous dismutation of superoxide radicals and thus reduces the level of superoxides. In response to the increased production of ROS followed by the oxidative damage to the neuron, the concentrations of antioxidant enzymes may increase as a compensatory process, thereby representing the most important endogenous defense against oxidative stress. However, as AD progresses, this defense is not sufficient and additional nonenzymatic antioxidant levels are most probably increased in order to cope with the AD insult. There are strong preclinical and clinical evidence on excessive free radical production and deficiency of antioxidant compounds in AD [148, 149].

Nuclear factor erythroid 2-related factor 2 (Nrf2) is a key transcription factor that regulates the functional expression of oxidative stress-related genes and derived endogenous antioxidants in response to ROS. During the oxidative damage insult, Nrf2 is translocated to the nucleus and binds to the antioxidant response element (ARE) in the promoters of antioxidant enzyme genes, which can subsequently enhance their protein expression, further contributing to the decrease of the oxidative stress insult [150]. The TCMs owing a large number of phenolic hydroxyl groups are natural strong antioxidants for detoxifying ROS and restoring mitochondrial membrane potential [151]. Artemisinin and analogs protected the HT-22 mouse hippocampal cell cultures from glutamate-induced oxidative damage [49]. It was also reported that Artesunate restored redox balance in LPS-induced inflammatory responses in microglial cells by inducing the activation of Nrf2-ARE signaling followed by increased expression of the downstream antioxidant enzyme, heme oxygenase-1 (HO-1) [62, 152]. Artemether caused activation of Nrf2 signaling, conferring neuroprotection towards A*β*-induced neurotoxicity in a 3xTg AD mouse model [59]. Ginsenoside Re attenuated A*β*-evoked ROS production, inhibited mitochondrial apoptotic pathway, and activated Nrf2-antioxidant response in A*β*-insulted SH-SY5Y neuroblastoma cell cultures [153]. Ginsenoside CK was found to enhance memory function, normalize neuronal morphology, decrease neuronal apoptosis, increase SOD and GpX levels, reduce malondialdehyde lipid peroxidation levels, inhibit A*β* expression, and activate the Nrf2 signaling pathway in a model of scopolamine-induced, memory-impaired mice [154]. Ginsenoside Rb-1's neuroprotective effects on memory and cognitive function in Alzheimer's disease rats were correlated with reduced apoptosis of hippocampal neurons and upregulation of the expression of antioxidant Nrf2, HO-1, and NAD(P)H quinone dehydrogenase-1 (NQO1) genes, increasing the activities of CAT, GSH, and SOD protein enzymes [155]. Ginsenoside F1, the metabolite of ginsenoside Rg1, repaired hippocampal long-term potentiation and memory in the APPswe/PSEN1dE9 AD mouse model, in correlation with increased activity of the antioxidant enzymes GpX and SOD [156]. In *in vitro* experiments using neuronal cultures, Astragaloside IV (AS-IV) improved cell viability by reducing apoptosis and decreasing the generation of ROS and mitochondrial superoxide induced by A*β*_1-42_. Furthermore, AS-IV inhibited the mitochondrial permeability transition pore opening, corrected the loss of mitochondrial membrane potential, and enhanced ATP level, thereby reducing cell death induced by mitochondrial dysfunction [157]. More recently, it has been found that AS-IV treatment of AD transgenic mice alleviated iron overload, by reducing oxidative stress [158].

### 4.3. Correction of Mitochondrial Dysfunction

Mitochondrial dysfunction leading to neuronal apoptosis is thought to be an early event in the development of AD. It is therefore important to target mitochondrial dysfunction in the early phase of AD to slow or prevent the neurodegenerative process and restore neuronal function [159]. Current research suggests that TCM by correcting mitochondrial reduced ATP level, membrane potential and calcium are conferring neuroprotection, thereby inhibiting PCD as reflected by the decrease in the level of the key signal molecules of mitochondrial apoptosis pathway, such as Bcl-2, Bax, Cyt-C, and caspase-3. For example, Artemisinin protected PC12 cells towards A*β*-induced damage in PC12 cells, by restoration of the mitochondrial membrane potential and inhibition of caspase 3/7 activity [56]. Similarly, Artemisinin pretreatment of SH-SY5Y neuroblastoma cells attenuated A*β*_1-42_-induced apoptosis by restoring the mitochondrial membrane potential and the levels of Bcl-2, Bax, cytochrome c, cleaved caspase-3, and cleaved caspase-9 [55]. Bilobalide, the main constituent of the nonflavone fraction of EGb761, was able to reduce p53, Bax, and caspase-3 protein expression as well as to inhibit apoptosis in PC12 cell cultures treated with a ROS inducer [160]. EGb761 neuroprotective action towards A*β*-induced damage was investigated in human neuroblastoma cell cultures indicating inhibition of ROS accumulation, mitochondrial dysfunction, and PCD [161]. EGb761 antioxidant properties have been attributed to its flavonoid fraction responsible for the direct ROS scavenging, prooxidant transitional metal ion chelation, and upregulation of SOD and GSH activities. Similar to EGb761, ginkgolide B improved mitochondrial function [162].

## 5. TCMs Modulate Neuroprotective Signaling Pathways

### 5.1. TCMs Activate Wnt/*β*-Catenin

Increasing evidence suggests that the pathological inactivation of the Wingless-related integration site protein (Wnt)/*β*-catenin signaling pathway is closely related to the occurrence and development of aging-related neuronal disorders such as AD [163].Wnt/*β*-catenin signaling is fundamental for neuronal survival and stem cell neurogenesis and is involved in the regulation of synaptic plasticity and BBB integrity and function. This signaling pathway is inhibited in the brain of AD patients, and its activation suppressed A*β* production and tau protein hyperphosphorylation [164]. Therefore, the use of TCMs to activate Wnt/*β*-catenin signaling provides a promising approach for the treatment of AD and other aging-related disorders. Notoginsenoside R1 (NGR1), one of the main effective components of *Panax notoginseng*, promotes growth of cultured cortical neurons from the neonatal rat, via the Wnt/*β*-catenin signaling pathway [165] and conferred neuroprotection towards glutamate-induced neurotoxicity in HT22 hippocampal neuronal cell cultures by upregulating the SIRT1/Wnt/*β*-catenin pathway [166]. Ginsenoside Rg1 conferred neuroprotection in both in vivo and in vitro models of Parkinson's disease through the Wnt/*β*-catenin signaling pathway [167]. Interestingly, Astragaloside IV exerted cognitive benefits and promoted hippocampal neurogenesis in a stroke mouse model by downregulating the proinflammatory cytokine interleukin-17 expression via activation of Wnt signaling pathway [168]. *Ginkgo biloba* extract and Ginkgolide B promoted neuronal differentiation of neuronal stem cells derived from the mouse brain postnatal subventricular zone and increased the nuclear level of *β*-catenin and activated the canonical Wnt pathway [169], and bilobalide promoted neuronal differentiation through activation of the Wnt/*β*-catenin signaling pathway [170]. These cumulative findings propose the involvement of the Wnt/*β*-catenin signaling pathway in the therapeutic effect of TCMs on brain injuries and neurodegenerative disorders such as AD (Figure 1(e)).

### 5.2. TCMs Modulate the PI3K/Akt/ mTOR Signaling Pathway

The PI3K/AKT signaling pathway is an important regulatory phosphorylation pathway in the central nervous system triggered by diverse stimuli, including neurotrophins, growth factors, cytokines, and cellular stress, that controls neuronal survival by both transcription-dependent and transcription-independent effects [171]. This pathway also links AD cellular processes such as amyloid-*β*, neurofibrillary tangles, and brain atrophy. The PI3K-Akt pathway regulates various biological processes such as cell survival, proliferation, motility, growth, survival, metabolic functions, synaptic plasticity, and neurogenesis and inhibits many neurotoxic mechanisms [172]. PI3K-Akt phosphorylates and regulates many transcription factors (CREB, NF*κ*B), and a large variety of cellular functions such as protein synthesis (4E-BP1, S6K), autophagy (mTORC1), cell survival (Bad), cell cycle progression (cyclin-D1, p21, and p27), cell differentiation, apoptosis (FoxO1, Bim, Bax, Bcl-2, and p53), angiogenesis (HIF-1), cerebral blood flow (eNOS), enzymes implicated in glucose metabolism (GSK-3, hexokinase, and ATP-citrate lyase), and expression and trafficking of glucose transporters [173]. The involvement of PI3K-Akt signaling in mitochondrial aerobic respiration has general important implications on oxidative stress insult contributing to AD [57]. Therefore, disruption of PI3K/AKT-mediated signal transduction significantly contributes to the pathology of AD [174] and represents a target of TCMs for therapy of AD [175]. The mammalian target of rapamycin (mTOR) is a highly conserved serine-threonine kinase that is activated in response to various upstream signals such PI3K/Akt phosphorylation and mediates tau phosphorylation, representing a risk factor for Alzheimer's disease [176]. Glycogen synthase kinase-3 (GSK3) is a serine/threonine kinase substrate of Akt, inhibited by Akt, that plays a key role in the pathogenesis of AD contributing to amyloid-*β* production, amyloid-*β*-mediated neuronal death, and hyperphosphorylation of microtubule-associated protein tau [177]. GSK3 inhibitors therefore show benefits in AD models of neurodegeneration [178]. Therefore, targeting and modulating the PI3K/AKT pathway activities and its downstream phosphorylated substrates have been proposed as a reasonable approach to confer neuroprotection and represent a common target of TCMs' beneficial effect in the treatment of AD [175, 179]. Consistent with this proposal, preclinical studies indicated that Artemisinin improved neuronal functions in Alzheimer's disease animal model 3xTg mice and neuronal cells via stimulating the ERK/CREB signaling pathway [62] while Artesunate promoted the proliferation of neural stem/progenitor cells by activation of the PI3K/AKT pathway [180]. Ginseng and ginsenoside Rg2 improved the memory ability and reduced the content of A*β*1-42 and p-tau in the AD rat model in correlation with PI3K/Akt signaling pathway activation [181, 182]. Ginsenoside Rd reduced A*β*-induced increased expression and activation of GSK-3*β*, attenuating A*β*-induced pathological tau phosphorylation in A*β*-treated cortical neuronal cultures and in a rat and transgenic AD mouse model [183], and inhibited mTOR activation in A*β*-treated PC12 cell cultures [184]. Astragaloside IV targeted PI3K/Akt [185] and conferred neuroprotection by activating the PI3K/Akt signaling pathway in the *in vitro* model of insulted PC12 neuronal cultures [186] and activated this pathway in blood vessel-derived endothelial cells [187]. *Ginkgo biloba* extract activated the PI3K/Akt/mTOR pathway in human and mouse neuroblastoma cell cultures, in correlation with suppression of the phosphorylation levels of tau [188, 189]. Activation of Akt by phosphorylation of Ser473 induced phosphorylation of tuberous sclerosis complex-2 (TSC2; phosphorylation at Ser 939) and inhibited its activity (TSC2 serves as a brake of mTOR) that in turn activates mTOR (phosphorylation at Ser 2448) inducing neuronal survival, neurite outgrowth, and neuroplasticity. In parallel, TCM inactivates GSK3*β* by increasing the phosphorylation of Ser 9 and thereby is blocking the antagonism on the Akt/mTOR pathway, amplifying the response [190]. Cumulatively, these examples indicate that TCMs in conferring neuroprotection in AD regulate by multiple mechanisms the balance of expression and protein phosphorylation of the PI3K/Akt/mTOR pathway (Figure 2).

### 5.3. TCMs Modulate MAPK Signaling Pathway

The signaling pathway of the microtubule-associated protein kinase (MAPK) which includes c-Jun N-terminal kinase (JNK), extracellular signal-regulated kinases 1 and 2 (ERK1/2), and p38 is increased in brain extracts of AD patients; chronically elevated levels of A*β* induce its dysregulation in the hippocampus and is a key element of the neuroinflammatory pathways triggered by glial cells during the development of AD [191, 192]. c-Jun N-terminal kinases (JNKs) show overactivation in AD brains and are responsible for the building-up of A*β* aggregates and tangles of tau protein [193]. Therefore, pharmacological mechanisms of TCM-induced neuroprotection address modulation of the MAPK signaling cascade [194], by preserving a balanced MAPK/ERK phosphorylation activity, which is an important approach in AD therapy [195] (Figure 3). The major compounds of ginseng oil attenuated A*β* 25-35-induced neuronal apoptosis and inflammation by modulating the MAPK/NF-*κ*B pathway in A*β*_25-35_-stimulated PC12 cell cultures [196]. In an in vitro study, ginsenoside Rb1 was shown to have a neuroprotective effect towards A*β*-induced damage in cultured hippocampal neurons by significantly increasing neurite outgrowth and stimulating the phosphorylation of extracellular signal-regulated kinase 1/2 (ERK1/2) [197]. AS-IV treatment reduced cortical neuron degeneration and memory deficits in AD rats by modulation of the ERK signaling [96]. EGb761 neuroprotective action towards A*β*-induced damage was investigated in human neuroblastoma cell cultures indicating inhibition of ROS accumulation, mitochondrial dysfunction, and PCD that were in direct correlation with the activation of c-Jun N-terminal kinase (JNK) and ERK 1/2 [161]. EGb761 increased autophagic activity and degradation of phosphorylated tau, in correlation with inhibition of p38-MAPK in human P301S tau mutant-transgenic mice [106]. These studies exemplify the beneficial modulatory abilities of TCMs on MAPK/ERK signaling in AD models.

### 5.4. TCMs Modulate the AMPK/GSK3*β* Signaling Pathway

AMP-activated protein kinase (AMPK) plays a major role in regulating cellular energy balance and may have broad neuroprotective effects in AD by promoting PCD autophagy, maintaining the control of the mitochondrial functions and relieving the oxidative stress insult [198]. Familial AD mutants of A*β* precursor protein and presenilin signal, at least in part, through the GSK*β* pathway [199] and tau protein undergo GSK*β*-mediated phosphorylation, resulting in decreased affinity of binding to the microtubules [200] and consequent neuronal cytoskeleton collapse and axonal transport impairment [201], thus contributing to the AD pathophysiology. Therefore, AMPK and GSK*β* represent potential therapeutic targets in AD therapy. Artemether modulation of AMPK/GSK3*β* signaling conferred neuroprotection towards A*β*-induced neurotoxicity in the 3xTg AD mouse model [60]. Ginsenoside Rb1 attenuated A*β*_25-35_-induced tau protein hyperphosphorylation in cortical neurons by inhibiting the expression of GSK-3*β* [202]. Ginkgolide B protected against A*β*_1-42_-induced apoptosis by activating the AMPK signaling pathway in rat astrocytes [203]. Egb761 attenuates zinc-induced tau phosphorylation at Ser262 by inhibiting GSK3*β* activity in rat primary cortical neurons [204], and bilobalide neuroprotective effects were associated with inhibition of GSK3*β* and reduction in A*β* levels [205].

## 6. Reducing Inflammation

Inflammation due to protein misfolding is one of the main pathological features of AD. Brain microglia cells play an important role in AD progression and a series of receptors expressed by these cells is involved in pattern recognition, A*β* oligomer and tau tangle clearance, and cellular activation [206]. So far, eight microglia innate immunity-related danger-sensing/pattern recognition receptors (PPRs) were found to respond to A*β* in the brain, and four of them activate microglia cells after A*β*-binding, promoting the activation of downstream inflammatory signaling cascades and ultimately causing neuronal damage [207]. These include the receptor for advanced glycosylation end products (RAGE), Toll-like receptors (TLRs), NOD-like receptors (NLRs), and progesterone receptor membrane component-1(PGRMC1/Sigma-2 receptor) [208]. The activation of transcription factor nuclear factor-*κ*B (NF-*κΒ*) regulates immune and inflammatory processes in response to A*β* lesions in the brain [209]. RAGE and TLR contribute to neuroinflammation by nuclear factor-kB (NF-kB) upregulation, promoting the expression of proinflammatory cytokines to induce a prolonged activation and promotion of signaling mechanisms for cell damage [210]. Activated microglia, astrocytes, and neurons release these inflammatory mediators and mediate neuroinflammation and neurodegeneration in a vicious manner. Further, immune and inflammatory cells and inflammatory mediators from the periphery cross the blood-brain-barrier and augment the neuroinflammation in AD [211]. Artemisinin and its analogs can effectively treat inflammation [212]. Artesunate significantly inhibited the release of proinflammatory mediators TNF*α* and IL-6 in BV2 mouse microglia-derived cell cultures exposed to LPS insult [57, 58]. *Gingko biloba* extract was found to improve cognitive function and decrease neuroinflammation and ameliorate the loss of synaptophysin in tau-transgenic mice and neuronal cultures [106]. Ginsenoside Rb1's neuroprotective effect has also been explored, with evidence suggesting its ability to revert the learning and memory impairments induced by A*β*_1-42_ intraventricular injection in correlation to suppressed expression of the neuroinflammatory markers in the hippocampus [213]. In addition, ginsenoside Rd alleviated the neuroinflammation [78]. TCM reduced inflammation by targeting and inhibition of the PPRs.

### 6.1. TCMs Inhibit RAGE

In general, natural compounds found to target RAGE, thereby reducing neuroinflammation, include iridoid glycosides, saponins, alkaloids, flavonoids, and polyphenols [214]. With this background and considering the selected TCMs addressed in this review, it is important to notice that Artesunate has proven its beneficial effects against ischemia/reperfusion injury in diverse organs, in direct correlation with its inhibition of RAGE, to inactivate the transcription factor NF-*κ*B and reduce the production of the proinflammatory cytokines IL-1*β*, IL-18, IL-6, and TNF-*α* [215]. However, to the best of our knowledge, this property of Artesunate or Artemisinin was not yet evaluated in preclinical AD *in vitro* and/or *in vivo* models. *Panax ginseng* enhanced significantly the learning and memory ability of AD' rats and attenuated oxidative stress damage by also blocking RAGE/NF-*κ*B activation [216]. Similarly, Astragaloside IV prevented memory impairment in D-galactose-induced aging rats via the AGEs/RAGE/NF-*κ*B axis [217]. *Ginkgo biloba* extract EGb761 induced clearance of A*β* by regulating RAGE expression in cerebral microvascular endothelial cells under chronic hypoxia and hypoglycemia [218] and reduced the A*β*-induced upregulation of RAGE in an in vitro bEnd.3, an immortalized mouse cerebral microvessel endothelial cell line model [219]. In line with these studies, *Ginkgo biloba* extract protected against chronic cerebral hypoperfusion by modulating RAGE-induced neuroinflammation in a rat model of bilateral common carotid artery occlusion [220]. Cumulatively, these studies may suggest that different TCMs, by common mechanisms of action, affect selectively a single or multiple cellular targets that are involved in inhibition of RAGE/NF-*κ*B activation (Figure 1(e)), resulting in decreased microglia-induced neural inflammation.

### 6.2. TCMs Inhibit TLRs

In general, natural compounds that were repeatedly reported to target TLRs and therefore alleviate chronic inflammatory response in AD include terpenoids, flavonoids, alkaloids, and coumarins [221]. Addressing the selected TCMs in this review, it is important to mention that Artesunate's beneficial effects were correlated with the inhibition of TLR4/MyD88/TRAF6 and thereby inactivation of the transcription factor NF-*κ*B and the production of proinflammatory cytokines [215]. Artemisinin B improved learning and memory impairment in AD mice with dementia by suppressing neuroinflammation by reducing the gene expression levels of MyD88 and NF-*κ*B as well as by reducing the protein levels of TLR4 and MyD88 [53]. *Panax ginseng* extract and ginsenoside Rg1 significantly suppressed the signaling transduction pathway of TLR3 and TLR4 and decreased the inflammation factors induced by A*β*_25-35_ in neuroglial NG108-15 cell culture [222]. Astragaloside IV exerted anti-inflammatory effects on microglia by inhibiting TLR4/NF-*κ*B signaling pathways and protected neurons from microglia-mediated cell death through microglia polarization [223]. Ginkgo diterpene lactones alleviated LPS-induced inflammatory response in primary astrocytes by downregulation of the TLR4/NF-*κ*B signal pathway [224], and ginkgolide B alleviated learning and memory impairment in rats with vascular dementia by reducing neuroinflammation due to decreased activity of the TLR4/NF-*κ*B pathway [225]. Cumulatively, these studies may indicate that the different selected TCMs presented here significantly reduced neuroinflammation and improved neuronal survival by reducing the secretion of inflammatory cytokines via downregulation or inhibition of the TLR4/NF-*κ*B pathway (Figure 1(e)), thus alleviating neurodegeneration in AD.

### 6.3. TCMs Inhibit NLRs

The nucleotide-binding oligomerization domain-like receptor- (NLR-) P3 (NLRP3) microglial inflammasome is a critical factor in stimulating innate immune responses, thus sustaining chronic inflammation. Therefore, targeting the NLRP3 inflammasome and the associated receptors could be a novel pharmacological strategy for development of TCM-like, anti-AD drugs, since its inhibition would selectively reduce AD chronic neural inflammation. Artemisinin significantly decreased amyloidogenesis and neuroinflammation in APPswe/PS1dE9 transgenic AD mice by mechanisms involving the suppression of the NALP3 inflammasome activation [226]. Ginseng saponins, including ginsenosides, alleviated inflammatory responses, and ginsenoside Rg3 suppresses the NLRP3 inflammasome activation through inhibition of its assembly [227–229]. Astragaloside IV attenuates cognitive impairments and reduced overactivation of microglia and the overexpression of inflammatory cytokines in the hippocampus, through its anti-inflammatory effects by inhibiting NLRP3 inflammasome overactivation [230]. More recently, it has been found that AS-IV treatment of AD transgenic mice alleviated iron overload, by reducing oxidative stress and inflammation [159]. *Ginkgo biloba* extract 50 (GBE50) inhibited the secretion of inflammatory factors after primary rat microglia activation, which was related to downregulation of the protein expression and activity of NLRP3 inflammasome [231], and ginkgolide B ameliorated hypoxic-ischemic brain injury in the neonatal male rat via inhibition of the NLRP3 inflammasome activation [232]. Cumulatively, these studies emphasize that part of the neuroprotective mechanisms of the selected TCMs presented here are mediated by anti-inflammatory effects, due to inhibition of the NLRP3 inflammasome overactivation in AD (Figure 1(e)).

## 7. Conclusions and Perspectives

The strength of this study is the analysis of preclinical and clinical evidences on the neuroprotective molecular and cellular mechanisms of selected TCM for AD therapy (Figure 1). It is difficult now to attribute the neuroprotective activity of a plant extract to a single compound or class of compounds as the observed beneficial properties are most probably the result of synergistic effects between multiple compounds and multiple pharmacological targets. The compounds of TCM presented here are lactones (Artemisinin, ginkgolides, and bilobalide), glycosides and triterpenoid saponins (ginsenosides, Astragaloside IV), and flavone glycosides (Ginkgo quercetin) that incorporate saturated and aromatic ring systems and chiral centers in their structures, contributing to a chemical diversity and structural complexity. The well-characterized pathological features of AD, including extracellular plaques of amyloid-beta and intracellular hyperphosphorylated fibrillary tangles of tau protein, induce calcium overload, oxidative stress, decreased cholinergic functions, and excitotoxic cell death and instigate an abnormal PCD cascade in susceptible brain regions (cerebral cortex, hippocampus, etc.), dysregulating the neuronal organelles (mitochondria and endoplasmic reticulum) and major signaling pathways such as Wnt/*β*-catenin, PI3K/AKT/mTOR, AMPK/ GSK-3*β*, and MAPK. This dysregulated PCD cascade ends with an abnormal neuronal loss which is a primary event that may precede the other events of AD neurodegeneration and that well correlates with the degree of dementia. The TCM presented in this review corrected the PCD cascade by a wide variety of neuroprotective antioxidative and anti-inflammatory mechanisms (Figure 1), in line with similar findings for other phytochemicals derived from natural plants such as Curcuma [233, 234] and Mucuna pruriens [235, 236]. Curcuma, for instance, contains high concentrations of polyphenols and flavonoids, and Mucuna contains tannins, polyphenols, and alkaloids, all conferring neuroprotection in different neurodegenerative disease models such as Parkinson's disease, Alzheimer's disease, amyotrophic lateral sclerosis, and ischemic stroke. The ability of the TCM reviewed here to confer neuroprotection towards the above PCD cascade in AD preclinical models (Figure 1(e)) may be valuable and advantageous in developing potential therapeutics for the treatment of AD. The efficacy of these TCMs in therapy of preclinical AD animal models and the promising exploratory clinical results propose their examination in patients with Alzheimer's disease in carefully designed clinical trials. In order to develop promising new TCMs, there is a need for a deeper understanding of the AD markers, establish a strong link between treatment targets, improve the translational measures, select the most promising investigational compounds, and improve clinical study design, in addition to the sharing of ideas, information, and knowhow on the progress in AD treatment across the Western world and Asia [237].

An important aspect that may limit the therapeutic applications of these TCM for AD therapy is related to their low solubility, short half-life, and poor bioavailability [238]. To increase bioavailability, reduce metabolic degradation, and improve the transfer through the blood-brain-barrier, new pharmaceutical technologies are required such as micro- and nanoencapsulation [239, 240]. The dosage required for beneficial safe effects in humans and without adverse reactions and drug interactions with other drugs in use are also important factors to be taken into consideration that needs longitudinal investigations.

## Figures and Tables

**Figure 1:** Neuroprotection induced by Artemisia, Ginseng, Astragalus, and Ginkgo traditional Chinese medicines for the therapy of Alzheimer's disease. (a) Several Artemisinin analogs such as Artemether and Artesunate can attenuate A*β*25-35-induced cognitive impairments by downregulating A*β*, BACE1, and tau proteins in different AD mouse models. (b) Compounds of Ginseng which have a four-ring steroidal structure with attached sugar moieties that account for their pharmacological activities by enabling their interaction with cell membranes, ion channels, and receptors. (c) AS-IV is the main active ingredient in Astragalus. AS-IV treatment reduced cortical neuron degeneration and memory deficits in AD rats and inhibited A*β*-induced PD. (d) Ginkgo biloba extracts can reduce the A*β* toxicity by inhibiting the formation of A*β*-fibrils, and ginkgolide A, bilobalide, and flavonoids can enhance the degradation of the phosphorylated-cytoskeleton tau protein in the lysosomes of neurons. In addition, Gingko biloba extract can improve cognitive function, decrease phosphorylated-tau protein levels, and ameliorate the loss of synaptophysin in tau-transgenic mice and neuronal cultures. (e) Calcium overload, mitochondrial dysfunction, and oxidative cell injury induced by misfolded tau and *β*-amyloid play an important role the pathological changes seen in AD. Red arrows indicate increase and blue arrows indicate decrease of signals, all contributing to neuroprotection in AD.

**Figure 2:** The neuroprotective effect of TCMs on AD through protein phosphorylation by the PI3K/Akt/mTOR pathway. Artemisinin, Astragaloside IV, ginsenoside Rb1, and 20(s)-protopanaxadiol activated PI3K/Akt kinases which in turn blocked downstream the activation of GSK-3*β* and reduced the content of p-tau in AD.

**Figure 3:** TCM-induced neuroprotection by modulation of the MAPK/ERK signaling. Artemisinin, ginsenoside Rb1, and Astragaloside IV from TCM activate the ERK1/2 phosphorylation and preserve a balanced MAPK/ERK phosphorylation activity contributing to a decrease amount of A*β* aggregates and tangles of tau protein in the brain of AD patients.
